The article "Effect of sagittal femoral component alignment on biomechanics after mobile-bearing total knee arthroplasty" was retracted in 2021. Reason: plagiarism.

# Effect of sagittal femoral component alignment on biomechanics after mobile-bearing total knee arthroplasty

**DOI:** 10.1186/s13018-019-1458-5

**Published:** 2019-11-28

**Authors:** Yong-Gon Koh, Jin-Ah Lee, Hwa-Yong Lee, Dong-Suk Suh, Hyo-Jeong Kim, Kyoung-Tak Kang

**Affiliations:** 1 Joint Reconstruction Center, Department of Orthopaedic Surgery, Yonsei Sarang Hospital, 10 Hyoryeong-ro, Seocho-gu, Seoul, 06698 Republic of Korea; 2 Department of Mechanical Engineering, Yonsei University, 50 Yonsei-ro, Seodaemun-gu, Seoul, 03722 Republic of Korea; 3 Department of Sport and Healthy Aging, Korea National Sport University, 1239 Yangjae-dearo, Songpa-gu, Seoul, 05541 Republic of Korea

**Keywords:** Total knee arthroplasty, Mobile-bearing, Malalignment, Finite element analysis

## Abstract

**Background:**

Recently, there has been increasing interest in mobile-bearing total knee arthroplasty (TKA). However, changes in biomechanics with respect to femoral component alignment in mobile-bearing TKA have not been explored in depth. This study aims to evaluate the biomechanical effect of sagittal alignment of the femoral component in mobile-bearing TKA.

**Methods:**

We developed femoral sagittal alignment models with − 3°, 0°, 3°, 5°, and 7°. We also examined the kinematics of the tibiofemoral (TF) joint, contact point on the TF joint, contact stress on the patellofemoral (PF) joint, collateral ligament force, and quadriceps force using a validated computational model under a deep-knee-bend condition.

**Results:**

Posterior kinematics of the TF joint increased as the femoral component flexed. In addition, contact stress on the PF joint, collateral ligament force, and quadriceps force decreased as the femoral component flexed. The results of this study can assist surgeons in assessing risk factors associated with femoral component sagittal alignment for mobile-bearing TKA.

**Conclusions:**

Our results showed that slight flexion implantation may be an effective alternative technique because of its advantageous biomechanical effect. However, excessive flexion should be avoided because of potential loosening of the TF joint.

## Introduction

Mobile-bearing total knee arthroplasty (TKA) was developed in the 1970s as an alternative to fixed-bearing TKA to provide high conformity and low contact stress between the metallic component and the polyethylene (PE) insert [1–3]. Mobile-bearing TKA features full or partial conformity of the superior surface of the insert with femoral condylar geometry, while the inferior surface of the insert is flat to allow rotation or sliding on the tibial baseplate with minimal friction [4]. Conformity with mobility in mobile-bearing TKA allows both minimal contact stress and minimal constraint, which cannot be achieved in fixed-bearing TKA [4]. Moreover, the shear forces on the bone-implanted components are expected to be minimized with an associated smaller risk of tibial component loosening as well as with a higher resistance by the ligaments [5]. The associated potential risk of wear on superior and interior surfaces has been controversial in recent retrieval studies [6, 7]. Early positive results have been observed in the design of numerous mobile-bearing prostheses [6, 8]. The number of prosthetic designs differs in terms of the degree of conformity between the femoral and the bearing components, and the degree of constraint of the bearing on the tibial baseplate [5]. Several clinical studies have shown that postoperative range of motion is statistically related to preoperative range of motion and that a preoperative flexion may be a critical factor in causing postoperative flexion [9, 10].

The article "Effect of sagittal femoral component alignment on biomechanics after mobile-bearing total knee arthroplasty" was retracted in 2021. Reason: plagiarism.

Malalignment of the femoral or tibial components have been known to cause chronic pain, potentially developing into arthrofibrosis. Considering the femoral component, malalignment may even lead to patellar instability, ligamentous instability, and disturbed functional joint kinematics [11–13]. The advantage of self-alignment is that it accommodates tibiofemoral (TF) malalignment by using a mobile tibial insert that self-aligns depending on the femoral component in mobile-bearing arthroplasty. This has not yet been confirmed experimentally [14–16]. To avoid notching the femoral component can be anteriorly implanted in a component with an extended position. In a distal femur cutting in the flexed position, the femoral component can be located in the posterior direction to avoid anterior gap between bone and prosthesis [17]. A previous study has stated that each increase of 2° in the sagittal flexion of the femoral component led to a decrease of 1 mm in the flexion gap [18]. However, there has been no study that evaluates mobile-bearing TKA with respect to femoral component sagittal malalignment.

This study aims to investigate the biomechanical effect of femoral component sagittal malalignment in mobile-bearing TKA. We developed models with sagittal alignments of − 3°, 0°, 3°, 5°, and 7°. TF kinematics, TF contact point, patellofemoral (PF) contact stress, collateral ligament force, and quadriceps force were investigated under a deep-knee-bend condition. We hypothesized that the biomechanical effect will be positive under slight flexion.

## Materials and methods

### Computational knee joint model

In this study, we used the previously developed and validated finite element (FE) model [19–22]. A three-dimensional (3D) non-linear FE model for normal knee joint was developed using medical imaging data. The subject’s medical history showed no musculoskeletal disorders or related diseases arising from a malalignment in the lower extremity, which indicated a healthy knee joint. The model includes bony structures of the knee joint with soft tissues in the patellofemoral and tibiofemoral joint. The model was developed using computed tomography (CT) and magnetic resonance imaging (MRI) (Fig. 1). CT image was performed with 0.1 mm slice thickness using a 64-channel CT scanner (Somatom Sensation 64, Siemens Healthcare, Erlangen, Germany). MRI image was performed on a 3-T MR system (Discovery MR750w®, GE healthcare, Milwaukee, WI, USA) with GEM Flex-Medium coil. MRI scans were obtained with 0.4 mm slice thickness in the sagittal plane. The reconstructed CT and MRI models were combined in an appropriate alignment using a commercial software (Rapidform version 2006; 3D Systems Korea Inc., Seoul, South Korea). Bones were assumed to be rigid because bone stiffness is much higher than that of the relevant soft tissues, and its influence in this study was negligible [23]. The major ligaments were modeled with nonlinear and tension-only spring elements [24, 25]. The ligament insertion points were determined with respect to the anatomy seen in the magnetic resonance imaging of the subject and descriptions based on previous studies (Fig. 1) [26–28].

The article "Effect of sagittal femoral component alignment on biomechanics after mobile-bearing total knee arthroplasty" was retracted in 2021. Reason: plagiarism.

**Fig. 1:** Methodology for ligament insertion points using magnetic resonance imaging when developing intact knee joint 3D model

To develop models for the changes in femoral sagittal alignment, two experienced surgeons (the second and sixth authors) performed a surgical simulation of a TKA. The simulation was conducted using Unigraphics NX (Version 7.0, Siemens PLM Software, Torrance, CA, USA). Computer-assisted design models of a mobile-bearing TKA from LCS (Johnson & Johnson—DePuy Orthopaedics, Inc., Warsaw, IN, USA) were virtually implanted into the bone geometry. A large-sized femoral component and size 4 tibial baseplate for mobile-bearing TKA were selected based on the dimensions of the femur and tibia, respectively. In the neutral position, in aligning the components in the coronal plane, the femoral component was set perpendicular to the mechanical axis connecting the center of the knee and the center of the femoral head. The tibial component was set perpendicular to the mechanical axis connecting the center of the knee and the center of the ankle joint. The rotational alignments of the femoral and tibial components were positioned in line with the femoral epicondylar and tibial anteroposterior axes, respectively. To develop the femoral component sagittal alignment models, the femoral component was positioned at − 3°, 0°, 3°, 5°, and 7° flexion in the plane parallel to the anterior cortex of the distal femur in the different simulated implantations (Fig. 2). The thickness of the distal bone cut was equal to the thickness of femoral component’s distal condyle.

The article "Effect of sagittal femoral component alignment on biomechanics after mobile-bearing total knee arthroplasty" was retracted in 2021. Reason: plagiarism.

**Fig. 2:** Developed five mobile-bearing TKA models with **a** − 3°, **b** 0°, **c** 3°, **d** 5°, and **e** 7° of femoral component flexion in sagittal alignments

In the TKA, contact conditions were applied between the femoral component and the PE insert, between the femoral component and the patellar button, and between the tibial component and the PE insert. The coefficient of friction between the PE material and the metal was selected as 0.04 for maintaining consistency with the explicit FE models proposed in previous studies [29]. The femoral component, PE insert, tibial component, and bone cement were composed of a cobalt chromium alloy (CoCr), ultra-high-molecular-weight polyethylene (UHMWPE), titanium alloy (Ti6Al4V), and poly (methyl methacrylate) (PMMA), respectively [29–31]. The material properties for each TKA component are listed in Table 1. A cement layer with a constant penetration depth of 3 mm into the bone was considered. It was based on a test of different cementing techniques at the femoral and tibial resection surfaces that were in contact with the femoral and tibial components, respectively [32]. The interfaces between the prosthesis and the bone were rigidly fixed by the cement used in this study [31]. Convergence was defined to be a relative change of more than 5% between two adjacent meshes with a mean edge length of 1.2 mm [33]. The 15,302 elements were used to construct TKA model.

**Table 1:** Material properties for FE model

	Young’s modulus (MPa)	Poisson’s ratio
CoCr alloy	220,000	0.30
UHMWPE	685	0.47
Ti6AI4V alloy	110,00	0.30
PMMA	1940	0.4

### Loading and boundary conditions

The changes in the femoral sagittal alignment model topologies provided six degrees of freedom to the TF and PF joints. The FE investigation included two types of loading conditions that corresponded with the loads used in the experiments that studied the TKA model validation and model predictions under deep-knee-bend loading conditions. The intact model was validated in a previous study [19–22], and the TKA model was validated through a comparison with the models used in a previous study [34]. An anterior force of 133 N and posterior force of 89 N were applied to 30° and 75° flexions followed by a measurement of the total anterior-posterior (AP) displacement to validate the mobile-bearing TKA model under the first loading conditions [34]. The second loading conditions corresponded to a deep-knee-bend loading that was applied to evaluate the effects of the changes in femoral sagittal alignment. Computational analysis was performed with anterior-posterior force applied to the femur with respect to the compressive load applied to the hip with femoral internal-external rotation constrained, medial-lateral translation free, and flexion determined by a combination of vertical hip and quadriceps load, leading to a six degrees of freedom TF joint [35, 36]. A proportional integral-derivative controller was incorporated into the computational model to control the quadriceps in a manner similar to that in a previous experiment [37]. A control system was used to calculate the instantaneous quadriceps displacement that was required to match the target flexion profile and was the same as that used in the experiment. Internal-external and varus-valgus torques were applied to the tibia, with the rest of tibial degree of freedoms constrained [35, 36].

The article "Effect of sagittal femoral component alignment on biomechanics after mobile-bearing total knee arthroplasty" was retracted in 2021. Reason: plagiarism.

The FE model was analyzed using Abaqus FEA (formerly ABAQUS) software, Version 6.11 (Dassault Systèmes Simulia Corp., Johnston, RI, USA). The kinematics of the TF joint, PF contact stress, force in the collateral ligaments, and quadriceps muscle forces were calculated throughout the deep-knee-bend loading conditions. The AP TF joint translation was calculated based on Grood and Suntay’s definition of the joint coordinate system [38].

## Results

### Validation of mobile-bearing TKA model

In the FE model used for the TKA, the AP translations in the TF joint were 8.7 and 7.3 mm at 30° and 75° flexions, respectively (Fig. 3), which was in agreement with a previous study that used experiments within one standard deviation under identical loading conditions applied to the prosthesis [34].

**Fig. 3:** Comparison of AP translations in TF joint at 30° and 75° flexions between our computational model and previous experiment for validation of mobile-bearing TKA model

### Comparison of kinematic and contact point on TF joint and contact stress on PF joint

Figure 4 shows that kinematics of the TF joint changed as the femoral component flexed under deep-knee-bend activity. Posterior translation on the TF joint also increased with the increase in femoral component flexion (Fig. 4). FE models for mobile-bearing TKA showed posterior femoral rollback of their lateral condyle, while the medial condyle remained in a similar contact position during a deep-knee-bend condition (Fig. 5). However, the posterior position of the contact point was observed when the femoral component sagittal flexion increased in any angle of flexion during deep-knee-bend activity (Fig. 5). Contact stress on the PF joint decreased as the femoral component flexed during deep-knee-bend activity (Fig. 6). The 7° flexion model showed that contact stress on the PF joint decreased by 9.4% as compared to the − 3° model (Fig. 6).

The article "Effect of sagittal femoral component alignment on biomechanics after mobile-bearing total knee arthroplasty" was retracted in 2021. Reason: plagiarism.

**Fig. 4:** Comparison of kinematic on TF joint with − 3°, 0°, 3°, 5°, and 7° of femoral component flexion models in deep-knee-bend loading condition

**Fig. 5:** Contact point changes on TF joint with **a**− 3°, **b** 3°, and **c** 7° of femoral component flexion models at 0°, 30°, 60°, 90°, and 120° flexions

**Fig. 6:** Comparison of contact stress on PF joint with − 3°, 0°, 3°, 5°, and 7° of femoral component flexion models in deep-knee-bend loading condition

### Comparison of collateral ligament force and quadriceps force

Figure 7 shows collateral ligament force change as the femoral component flexed during deep-knee-bend activity. Both medial and lateral collateral ligaments’ forces decreased as the femoral component flexed. A similar trend was found in the quadriceps force (Fig. 8). It required the largest lumped quadriceps forces during deep flexion as the femoral component flexed. The flexion 7° model showed that the quadriceps force decreased by 10.4% compared to the − 3° model.

**Fig. 7:** Comparison of (**a**) medial and (**b**) lateral collateral ligament force with − 3°, 0°, 3°, 5°, and 7° of femoral component flexion models in deep-knee-bend loading condition

**Fig. 8:** Comparison of quadriceps force with − 3°, 0°, 3°, 5°, and 7° of femoral component flexion models in deep-knee-bend loading condition

## Discussion

A significant finding of this study was that an advantageous biomechanics effect occurred as the femoral component flexed. However, excessive flexion should be avoided because of the risk of progressive loosening of the TF joint.

Soft tissue conditions in mobile-bearing TKA play a considerably important role compared to fixed-bearing TKA [39]. One of the major goals of mobile-bearing TKA is to promote load-sharing through the relative displacement of the tibial and femoral components [39]. Soft tissue should be encouraged to decrease the dependency on intrinsic constraints owing to the condylar geometry. Therefore, information on soft tissue tension is indispensable for determining kinematics and clinical results following mobile-bearing TKA. However, there is a lack of soft tissue information in previous fluoroscopy studies. Moreover, each study has shown different results. Potential reasons for this difference may include different TKA designs, confounding variables such as soft tissue contractures that are difficult to control in-vivo, and sample size.

The article "Effect of sagittal femoral component alignment on biomechanics after mobile-bearing total knee arthroplasty" was retracted in 2021. Reason: plagiarism.

Many factors affect the postoperative range of motion. Previous studies have reported the effect of implant alignment and the relative position of the prosthesis on the postoperative range of motion [40, 41]. The plastic bone models that were used did not represent the variability that is typically present among subjects. However, this problem can be overcome by using a computational study. This is because computational simulation for a single subject has the advantage of determining the effects of the femoral component’s sagittal alignment position within the same subject and of eliminating the effects of other variables, such as the subject’s weight, height, bony geometry, ligament properties, and component size [42, 43].

In this study, we have evaluated the important variables that may determine the biomechanical effect in mobile-bearing TKA. The mobile-bearing TKA model was validated using experimental and kinematics data [34]. Therefore, the TKA model developed in the study is considered reasonable. Our results showed that posterior translation on the TF joint increased as the femoral component flexed. Posterior TF translation is important in TKA because it can provide greater flexion before TF impingement occurs [44]. The femoral component is implanted more posteriorly and more proximally, together with a more anterior tibial insert located with a femoral component flexion. In other words, late TF impingement could occur as the TF joint posterior translation increased in femoral component flexion, and range of motion may increase.

The TF joint contact point supported this result. Several studies have used in-vivo weight-bearing fluoroscopy to evaluate TF kinematics after TKA. A previous study evaluated the lateral condylar motion of TKAs using a 3D inverse perspective technique during a deep-knee-bend activity, and found that the lateral condyles began slightly anterior to the midline of the tibial sagittal plane in extension and had posterior femoral rollback with flexion similar to normal knees [45]. The researchers reported an average posterior femoral rollback of 7.7 mm, with the highest amount being 12.3 mm [45]. Another previous study evaluated mobile-bearing TKA with the same fluoroscopic technique and analysis and found that the implant showed minimal rollback from 0° to 60° flexion followed by mild anterior translation with increased knee flexion [46]. All TKAs were noted to start posterior to the sagittal midline at full extension.

In the current study, a computational model of mobile-bearing TKA showed a contact position near the midline tibia in extension. It is similar to the trend shown in a fluoroscopic study using the same TKA as that used in this study [47]. Our computational model’s anterior slide of the femoral component occurred at either 30° or 60° knee flexion during deep-knee-bend activity. Our model exhibited more posterior femoral rollback of the lateral condyle, which leads to achieving normal axial rotation patterns. The LCS implant has high conformity to 30° flexion, which shows a relatively neutral positioning in extension. Femoral geometry changes on the posterior condyles with a diminishing radius of curvature lead to the tendency toward anterior translation in deeper flexion. Similar to posterior cruciate retaining TKA that experiences anterior translation as flexion increases, this movement may cause extensor mechanism deficiency and diminished range of motion [47]. However, a previous study showed a range of motion of 162° for Japanese subjects implanted with this TKA. In relation to articular wear and interface loading, the midline positioning for mobile-bearing TKA may be considered optimal [48]. Posterior TF translation is important in TKA because it provides higher degree of flexion prior to the occurrence of TF impingement [42, 49]. Our study showed increased posterior TF translation as femoral component flexed. It provides potential of higher degree flexion.

The article "Effect of sagittal femoral component alignment on biomechanics after mobile-bearing total knee arthroplasty" was retracted in 2021. Reason: plagiarism.

Our results showed that the quadriceps force and contact stress on the PF joint decreased as the femoral component flexed, because a more posterior TF contact point at full flexion improves the quadriceps moment arm, which has been associated with improved International Knee Society Function scores in TKA [50, 51]. Previous studies found more posterior TF contact point in-vivo and reduced quadriceps forces ex-vivo [52, 53]. In addition, such a trend can be found in mobile-bearing TKA that posteriorly positioned TF contact point provided a better functional activity [54]. Our results also showed that increased femoral component flexion can be expected to reduce the quadriceps force and the PF contact stress required for deep-knee-bend activity to some extent. Since osteoarthritis and TKA patients are suffering from quadriceps weakness, extension femoral component that increases the required quadriceps force could make for patients to kneel, squat, or rise from a chair more difficult [55].

The study shows interesting results in terms of the collateral ligament. The collateral ligament force decreased as the femoral component flexed. Large amounts of sagittal femoral component extension may be harmful to the collateral ligament. Errors in femoral component sagittal alignment contribute to imbalanced soft tissue that leads to instability and a limited range of motion. However, this study showed that a more femoral component flexion loosens the TF joint in flexion. Interestingly, an increase in femoral component flexion produces remarkable effects in extension. This can be explained by translation of the femoral component flexion to all points of the tibial plateau distally, which loosens the TF joint throughout the entire knee flexion extension range. In clinical practice, if the extension gap has already been successfully balanced, any further increase in the femoral component flexion alters the level of the TF joint line, which reduces the force of the collateral ligament and increases the laxity of the knee both in flexion and in extension [56]. Such a trend can also be found in increased posterior tibial slope in which a contact point can be positioned posteriorly [42, 54]. In fact, there has been no information for collateral ligament force because excessive collateral ligament may cause ligament rupture and decreased collateral ligament may lead to TF joint loosening.

The article "Effect of sagittal femoral component alignment on biomechanics after mobile-bearing total knee arthroplasty" was retracted in 2021. Reason: plagiarism.

As mentioned previously, proper femoral component alignment is strongly related to greater stability, a lower rate of loosening, and higher clinical scores [11–13, 57, 58]. A previous study focused only on varus-valgus and internal-external rotation in the femoral component. However, our results showed that femoral component sagittal alignment, flexion-extension, may affect biomechanics. In a recent study, Antony et al. showed that the femoral component angle demonstrated positive correlation with maximum flexion angle and range of motion [59]. Another study also showed that slight flexion implantation may be an effective alternative technique to prevent excessive component overhang, especially in the trochlea and anterior region of the distal condyle, in patients with TKA [60]. Kim et al. studied the relationship between postoperative sagittal alignment of the femoral component and implant survival [61]. They stated that a femoral sagittal alignment of 0°–3° improved the survival rate of the knee prosthesis [61]. In addition, an advantage is the reduction of risk in femoral notching with the anterior bone cut as the femoral component is flexed [62, 63].

In terms of clinical relevance, the optimal femoral component sagittal angle should help surgeons cut the distal femur properly on the sagittal alignment. In the present study, excessive femoral component flexion led to instability of the TF joint. Based on previous results and of this study, we recommended slight flexion in the femoral component, while avoiding extension of the femoral component.

There are several limitations to this study. First, only one mobile-bearing prosthesis was used for the simulation; hence, our result cannot represent all mobile-bearing TKA. Second, this simulation was performed using a virtual and variable model, and the material properties for soft tissues referred to relevant cadaveric studies. These are common methods using a computational model. Third, because a standard computer simulation model was employed, neither statistical processing of the data nor calculation of standard deviations had to be performed. Finally, the results could not represent clinical outcomes and consider patient satisfaction because they corresponded to computational output. However, the main factor analyzed in the present study corresponded to the main investigated components to evaluate the biomechanical effect in computational biomechanics.

The article "Effect of sagittal femoral component alignment on biomechanics after mobile-bearing total knee arthroplasty" was retracted in 2021. Reason: plagiarism.

In conclusion, based on the results, the sagittal positioning of the femoral component is an important factor that affects knee joint biomechanics. Therefore, surgeons should be aware that any error in distal femoral resection may lead to a negative effect on knee joint biomechanics. We recommend slight flexion in sagittal alignment and avoiding extension of femoral component.

## Data Availability

Not applicable.

## Abbreviations

3D: Three dimensional
AP: Anterior-posterior
CoCr: Cobalt chromium alloy
FE: Finite element
PE: Polyethylene
PF: Patellofemoral
PMMA: Poly (methyl methacrylate)
TF: Tibiofemoral
Ti6Al4V: Titanium alloy
TKA: Total knee arthroplasty
UHMWPE: Ultra-high-molecular-weight polyethylene
